# Optimization of the Transverse Electric Photonic Strip Waveguide Biosensor for Detecting Diabetes Mellitus from Bulk Sensitivity

**DOI:** 10.1155/2021/6081570

**Published:** 2021-11-26

**Authors:** Prasanna Kumaar S., Sivasubramanian A.

**Affiliations:** School of Electronics Engineering, Vellore Institute of Technology, Chennai 600127, India

## Abstract

Diabetes mellitus is a chronic metabolic condition that affects millions of people worldwide. The present paper investigates the bulk sensitivity of silicon and silicon nitride strip waveguides in the transverse electric (TE) mode. At 1550 nm wavelength, silicon on insulator (SOI) and silicon nitride (Si_3_N_4_) are two distinct waveguides of the same geometry structure that can react to refractive changes around the waveguide surface. This article examines the response of two silicon-based waveguide structures to the refractive index of urine samples (human renal fluids) to diagnose diabetes mellitus. An asymmetric Mach–Zehnder interferometer has waveguide sensing and a reference arm with a device that operates in the transverse electric (TE) mode. 3D FDTD simulated waveguide width 800 nm, thickness 220 nm, and analyte thickness 130 nm give the bulk sensitivity of 1.09 (RIU/RIU) and 1.04 (RIU/RIU) for silicon and silicon nitride, respectively, high compared to the regular transverse magnetic (TM) mode strip waveguides. Furthermore, the proposed design gives simple fabrication, contrasting sharply with the state-of-the-art 220 nm wafer technology.

## 1. Introduction

Diabetes mellitus causes kidney failure, stroke, heart attacks, eye blindness, and lower limb amputation [1]. The traditional method for monitoring diabetes mellitus is an analysis of glucose concentration in human blood samples and plasma separated from blood [2]. Another well-established method is using “test strips” of different companies available in the market which changes the colour of the strip based on the glucose concentration present in urine; it is also referred to as “glycosuria.” [3] The low and high blood glucose concentration level is called hypoglycaemia [4] and hyperglycemia [3]. In blood, the glucose concentration indicates very high as compared to the urine sample, the level of glucose is seen small in the range of 0 to 15 mg/dl, and glucose present in urine is identified as the “renal threshold of glucose (RTG).” [3]

Physically, a urine sample will change the surface tension, gravity, and refractive index due to the presence of glucose. The noninvasive sensing method (urine sample) applied to the evanescent field photonic waveguide have been studied extensively due to sensitivity over the refractive index of a sample. Other specific characteristics of label-free biosensing are resistance to electromagnetic interference, compact design, the potential to integrate to lab on a chip, etc. These sensors lead to significant developments in diagnosis, food safety management, pharmaceutical development, and monitoring of environmental hazards [5]. As an outcome, various resonant structures such as Mach–Zehnder interferometers (MZIs) [6, 7], ring resonators [8], and modal interferometers [9] are broadly used for biological and chemical sensing.

Silicon photonic biosensing technology provides a new opportunity to analyze glucose concentration present in urine with optimized waveguide structures [6]. The propagation velocity of the electromagnetic field is high when the biological molecules are present in the waveguide structure as compared to other environments such as air and water. The wavelength shifts due to light absorption in a waveguide structure through electromagnetic waves with biological molecules. The wavelength shift is easily detected and measured by the sensor and used further for label-free biosensing [5, 7].

This work aims at developing an optimized silicon and silicon nitride waveguide biosensor that can be easily fabricated and reconfigured. The structure is designed to detect spectral changes over the waveguide surface of silicon and silicon nitride due to high glucose concentration present in the urine sample. The silicon and silicon nitride waveguide design has advantages such as simple fabrication and a wide range of biological detection [8]. Silicon nitride waveguide increases sensor scalability when tight bends are introduced and there is less loss in complex design structures [9]. Although other types of waveguides such as slot waveguides [10] and rib waveguides are available, the purpose to use strip waveguide as the waveguide could be fabricated without a cladding region for biosensor applications using evanescent field sensing (Figure 1).

## 2. Materials and Methods

The main advantage of the silicon-on-insulator (SOI) strip waveguide is strong optical confinement in the core as all three sides of the waveguide are surrounded by a low-index (or) analyte. The design of the MZI waveguide is shown in Figure 2. Fabrication of the SOI waveguide in CMOS foundry line with top layer comprising 220 nm silicon strip waveguide on 2 *μ*m buried silicon oxide [10]. The design specification of the silicon and silicon nitride waveguide biosensor and analyte refractive index (RI) are shown in Table 1.

### 2.1. Silicon Nitride (Si_3_N_4_) Waveguide

The silicon nitride (Si_3_N_4_) strip waveguide platform used to design low-loss photonic integrated chip (<1 dB/cm), which is suitable for the biosensing environment in the wavelength range from 400 nm to 2350 nm and fabrication, is similar to the silicon-on-insulator (SOI) wafer scaling process [12]. Silicon-on-insulator waveguide provides loss due to absorption of biomolecules in the surface, compared to silicon nitride based on the sample, e.g., blood and urine. The Si_3_N_4_ material is commonly used as a substructure in the fabrication of photonic circuits. Si_3_N_4_ is usually developed with other composites, which exhibits stable electronic, chemical, and structural interfaces [13]. The first Si_3_N_4_ fabrication on films on SiO_2_ wafers for the propagation of optical wavelength in the visible spectrum (632 nm) was reported [14, 15]. In the 1980s, the optical propagation through the straight-line Si_3_N_4_ waveguide, which plays an important role to use the specific material as a functional device, was earlier done by Heideman E. A. [16], with a partly integrated Mach–Zehnder interferometer (MZI) for sensing array, where the two arms of the MZI were Si_3_N_4_/SiO_2_ waveguides.

A single-mode silicon waveguide structure was initially reported [13] with 1-2 dB/cm loss in early-stage transmission compared to the current state-of-the-art technology fabrication of the silicon-on-insulator waveguide loss of 0.3 dB/cm [14]. Silicon nitride waveguides are preferred as they offer low waveguide loss and are flexible in fabrication compared to silicon-on-insulator (SOI) waveguides. This sensor can be integrated into mobile phones in the future, so the device operates at low power levels.

Nonlinear optical properties of the silicon-based waveguide have the main disadvantage of the existence of two-photon absorption (TPA) related effects that limit the use of the device in low power levels, mainly decreasing the nonlinear optical performance of the system. Silicon nitride layers are accurately engineered to show a high nonlinearity of the Kerr effect with no two-photon absorption (TPA) related effects. The approach makes it possible to operate waveguides at low power levels. The nonlinear properties of the photonic waveguide are generally modelled by the parameter *Y* in the following equation [16]:

(1) $$\begin{array}{c} Y\left(\omega \right)=\frac{3\omega }{4\varepsilon_{0}c^{2}A_{eff}n_{eff}}, \end{array}$$

where *ε*_0 _ is the vacuum permittivity,  *n*_*eff*_ is the modal effective refractive index at wavelength or frequency *ω*, and *A*_*eff*_ is the effective area of the particular waveguide. The effective area for each waveguide structure will be using the following equation [17, 18]:

(2) $$\begin{array}{c} A_{eff}=\frac{a_{NL}\left(\int \int_{-\infty }^{\infty }S_{z}dxdy\right)}{\iint_{NL}S_{z}dxdy}, \end{array}$$

where *a*_*NL*_  is the cross section of the core area and *NL* is the integration of the nonlinear region. The electrical and magnetic fields of the waveguide properties were calculated in the lumerical finite difference method (FDM) solver. TPA can be kept minimal around a wavelength of 1550 nm, allowing high-power operation, which was usually avoided in the standard silicon-on-insulator waveguide. Using the optimized silicon nitride material composition, a nonlinear phase shift of *π* can be attained, making it suitable for implementing telecommunication wavelength for integrated photonic biosensing applications [19].

### 2.2. Modelling Approach

The 3D Maxwell equation is solved by the finite-difference time-domain (FDTD) numerical method [20–22]. The lumerical FDTD solution can efficiently calculate the interaction of light with the waveguide structure over wide bandwidths [23]. The fundamental transverse electric (TE) mode is analyzed in Lumerical Mode Solutions software to find the effective index and effective area. In the proposed waveguide structure, 220 nm high and 800 nm wide agrees with standard CMOS foundry [10]. At 1550 nm wavelength sweep, the presence of the analyte in the waveguide leads to an evanescent field up to 30 nm above the waveguide structure. The evanescent field of the transverse electric (TE) mode propagation in silicon and silicon nitride is shown in Figures 3(a) and 3(b). In Figure 3(b), due to high contrast, silicon nitride waveguide with TE field is high compared to silicon material. This provides a better evanescent field in the waveguide surface and enhances the sensitivity.

The TM mode is irregular at waveguide core top and bottom borders, while the TE mode is irregular at waveguide sidewalls. In the waveguide, it applies to an analyte on top of the waveguide, so TE can be used to get accurate bulk sensitivity over the core top; the waveguide dimensions are width *W* at 800 nm and height *H* at 220 nm. The proposed waveguide sensor uses TE_00_. Different types of grating couplers are available for TE_00_ to integrate with the sensor at a low cost.

### 2.3. Determination of the Refractive Index of Urine

The refractive index of urine with different samples is calculated using Snell's law equation:

(3) $$\begin{array}{c} \mu =\frac{\sin\;i}{\sin\;r}, \end{array}$$

where *i* is the angle of incidence and *r* is the angle of refraction.

The sample varies, respectively, to temperature and wavelength of the transmission spectrum. Reaction of the sample *R*_*s*_ is given by

(4) $$\begin{array}{c} R_{s}=\left(\frac{\mu^{2}-1}{\mu^{2}+2}\right)\left(\frac{1}{d}\right). \end{array}$$

The refractive index of the sample is defined by the ratio of the light velocity in air and the medium velocity. Both healthy and diabetic person urine samples were collected from age group 22–64 at Hyderabad Diagnostic Centre, Malakpet, Hyderabad, India. Samples were collected and kept under uniform temperature and processed within an hour to avoid any bacterial growth, and molecular properties are not affected. These samples were placed in Abbe's refractometer to get a respective refractive index of different samples [3].

### 2.4. Circuit Simulation

The waveguide platform has Mach–Zehnder interferometer (MZI) design. The main advantage of the MZI configuration is that it provides more design options to enable high sensitivity and choose the wavelength spectrum independently [24]. The MZI has two arms with different lengths: reference arm is 100 microns long and sensing arm is 1 mm long [25]. The MZI is the main building block in the silicon photonic waveguide structure; it has many different roles to play with a modification. MZI can be used as a wavelength multiplexer [26], demultiplexer [27], isolator [28], switch [29], sensor [30], etc. MZI consists of a splitter, a combiner, and two asymmetric waveguide arms: the reference arm and sensing arm use dielectric-based (SiO_2_ or Si_3_N_4_) waveguide on the silicon substrate. The specification is more suitable for biosensing applications [31]. MZI waveguide structure is placed with different glucose concentrations in urine samples. The wavelength of light passes through the photonic waveguide from the splitter to the reference arm and sensing arm. Combiner, on the other end, gets detected due to the evanescent field. The propagation of light varies, and there is a shift in the frequency response in the waveguide structure. Based on the refractive index of different glucose concentrations present in the urine sample, this paper uses Lumerical Mode Solutions for solving bidirectional eigenmode expansion and var FDTD and Lumerical INTERCONNECT for circuit simulation. The mesh structure used in the simulation is near to fabrication sensitivity [32].

### 2.5. Bulk Sensitivity

Real-world point-of-care systems involve incorporating a diverse set of functionalities on the chip, ranging from analyte-light interaction to electronic signal transmission. The silicon-on-insulator (SOI) platform brings the opportunity to implement such technologies, including high-sensitivity waveguides, possibly the best semiconductor devices, compatibility with CMOS circuitry, and the potential of bulk production and lower cost of production. The sensitivity of the sensor increases, and TE mode field provides high overlap over the waveguide structure. Due to the high mode field with the analyte, the change in the effective index in the cladding region (*n*_*eff*_) based on the change in the refractive index of the analyte or sample is *n*_*c*_, bulk sensing equation (5) [33]. The minimum concentration required for bulk sensing is 0.625 gm/dL.

(5) $$\begin{array}{c} S_{b}=\frac{\partial n_{eff}}{\partial n_{c}}\frac{RIU}{RIU}. \end{array}$$

## 3. Results and Discussion

The refractive index of different glucose concentrations present in the urine samples is from 1.332 to 1.340 [3]. The diabetes mellitus patient's refractive index is very high. Morning urine samples have taken the mean value of the refractive index ranging from 1.336 ± 0.0019, and some random samples' refractive index is 1.335 ± 0.0017 [3]. The refractive index of glucose concentration in urine is susceptible to the transmission spectrum.

The transmission spectrum of silicon on insulator shows that the wavelength sweep gives a possible change in the output waveform. The refractive index of high glucose concentration (RI: 1.347) of the output waveform peaks and, varies in silicon on insulator (Figure 4) and silicon nitride (Figure 5).

The effective index measures sensitive changes in the waveguide structure with a respective wavelength. The effective index of a silicon-on-insulator waveguide is shown in Table 2, and the effective index of the silicon nitride waveguide is shown in Table 3. By the analysis, bulk sensitivity area is calculated in the silicon-on-insulator and silicon nitride waveguide which effectively covers the urine sample on the surface of the sensor. The effective sensing area increases with respect to the material which increases the sensitivity of the sensor.

Evanescent field interaction with the high glucose concentration (RI 1.347) sample over the waveguide structure causes refractive index to change. The transverse electric loss is reported in Figure 6 on high glucose concentrations (RI: 1.347).

The change in the output wavelength spectrum for various levels of glucose concentration is present in the urine. By the proposed sensor waveguide structure with two different materials, silicon and silicon nitride, the changes can be detected.

The proposed silicon and silicon nitride waveguide sensor can be detected to sense average and low glucose concentration present in urine samples (Figure 7). From the standard laboratory setup, colour change in sample determines the level of glucose present in the urine. This method of measuring glucose is not efficient to detect hypoglycemia [4, 34]. The hypoglycaemia condition is a low glucose concentration level present in blood (40 to 60 mg/dl) [34]. The refractive index of hypoglycaemia in blood is 1.2 [4]. The authors previously worked on optimizing the photonic waveguide structure to detect diabetes mellitus from blood samples [35, 36].

The proposed biosensor can help detect both low glucose “hypoglycemia” and high glucose “hyperglycemia.” Due to the ongoing COVID-19 pandemic situation, it has become indispensable to use a noninvasive glucose sensing method compared to the traditional blood pinpricking method. Figures 4 and 5 show the peak in the 1550.80 nm transmission spectrum for high glucose concentration in a silicon-on-insulator waveguide. The peak transmission spectrum at 1550.89 nm for high glucose concentration in the silicon nitride waveguide is detected. When biological molecules interact with the wavelength spectrum, the velocity of the electromagnetic field is reduced; hence, the transmission loss at 1550.80 nm is less. The proposed silicon-on-insulator and silicon nitride have a similar geometry structure with different materials on a waveguide-based biosensor which can easily detect glucose present in the urine sample.

## 4. Conclusions

The output is error free without any laboratory setup for regular glucose monitoring using the non-invasive (urine) method without any other chemical reagents added. The silicon photonic waveguide biosensor can detect the variations in the transmission spectrum at 1550 nm from glucose concentration present in urine with the input refractive index. The bulk sensitivity of the proposed strip waveguide of silicon and silicon nitride is fairly high with TE polarization. The design is simple and flexible with a similar geometry structure for the silicon and silicon nitride waveguide thickness of 220 nm and width of 800 nm with a typical MZI sensing arm. The analysis clearly shows the bulk sensitivity can achieve more than 1.09 (RIU/RIU) and 1.04 (RIU/RIU) for silicon and silicon nitride with a standard geometry thickness of 220 nm as shown in Table 4. It is easier to fabricate and is considered to be used as a full-filled single-mode condition. Early detection prevents millions of people detect diabetes mellitus and from type 2 diabetes-related issues such as kidney failure, heart attack, blindness, and lower limb amputation based on a WHO report.

## Figures and Tables

**Figure 1:** Strip waveguide structure.

**Figure 2:** Mach–Zehnder interferometer waveguide structure for the sensor [11].

**Figure 3:** Mode propagation of wavelength on the waveguide structure. (a) TE polarization mode in the SOI waveguide. (b) TE polarization mode in the silicon nitride (Si_3_N_4_) wire waveguide.

**Figure 4:** Transmission spectrum of silicon on insulator (SOI) with different urine samples.

**Figure 5:** Transmission spectrum of silicon nitride (Si_3_N_4_) with different urine samples.

**Figure 6:** Transverse electric loss for the silicon and silicon nitride waveguide structure.

**Figure 7:** Transmission spectrum for hypoglycemic and normal urine.

**Table 1:** Design specifications of the proposed biosensor.

Design parameter	Values
Waveguide structure	Strip waveguide
Thickness	220 nm
Width	800 nm
Waveguide material	Silicon and silicon nitride
Wavelength of light	1550 nm to 1560 nm
Analyte structure	130 nm thick and 800 nm wide
Thermo-optical coefficients	295 K
RI of the analyte structure	According to the urine samples taken with different glucose concentrations [3]

**Table 2:** Refractive index and bulk sensitivity of the silicon-on-insulator waveguide.

Refractive index (RI) of urine	Effective index in silicon on insulator	Bulk sensitivity *S*_*b*_ (RIU/RIU)
1.335	1.464494	1.09699
1.336	1.464676	1.09631
1.337	1.464859	1.09560
1.338	1.465042	1.09494
1.341	1.465592	1.09290
1.347	1.466700	1.08860

**Table 3:** Refractive index and bulk sensitivity of the silicon nitride waveguide.

Refractive index (RI) of urine	Effective index in silicon nitride	Bulk sensitivity *S*_*b*_ (RIU/RIU)
1.335	1.388407	1.04000
1.336	1.388425	1.03920
1.337	1.388497	1.03851
1.338	1.388542	1.03777
1.341	1.388676	1.03555
1.347	1.388948	1.03114

**Table 4:** Waveguide sensitivity comparative analysis.

Waveguide structures	Bulk sensitivity *S*_*b*_
TM photonic wire	0.37 (RIU/RIU) [37]
TE slot waveguide	0.83 (RIU/RIU) [37]
TE photonic wire	0.16 (RIU/RIU) [37]
TE photonic SOI strip waveguide (this work)	1.09 (RIU/RIU)
TE photonic Si_3_N_4_ strip waveguide (this work)	1.04 (RIU/RIU)

## Data Availability

The data underlying the results presented in this paper are not publicly available at this time but may be obtained from the authors upon reasonable request. The data of urine samples are taken from S. I. Ahmad, “Studies on some biophysical aspects of human renal excretory fluid,” Ph. D. dissertation, Jawaharlal Nehru Technological University, 2010 [3].
